The article "Suppression of Long Noncoding RNA SNHG1 Inhibits the Development of Hypopharyngeal Squamous Cell Carcinoma via Increasing PARP6 Expression" was published in 2022. Journal: Evid Based Complement Alternat Med.

# Suppression of Long Noncoding RNA SNHG1 Inhibits the Development of Hypopharyngeal Squamous Cell Carcinoma via Increasing PARP6 Expression

**DOI:** 10.1155/2022/1562219

**Published:** 2022-07-05

**Authors:** Qian Chen, Xiao He, Bin Li, Jingjing Chen, Xuxia Tang

**Affiliations:** Department of Otolaryngology, The First Affiliated Hospital of Zhejiang Traditional Chinese Medical University, Hangzhou 310006, China

## Abstract

**Purpose:**

This study aimed to explore the function and molecular mechanism of long noncoding RNA Small Nucleolar RNA Host Gene 1 (SNHG1) in the development of hypopharyngeal squamous cell carcinoma (HSCC).

**Methods:**

Human HSCC cell line FaDu was used in this study. Cell viability and apoptosis were detected using CCK-8 assay and flow cytometry, respectively. Cell migration and invasion were measured by Transwell assay. The expression of PARP6, XRCC6, *β*-catenin, and EMT-related proteins (E-cadherin and N-cadherin) were determined using western blotting. Moreover, the regulatory relationship between SNHG1 and PARP6 was investigated. Furthermore, the effects of the SNHG1/PARP6 axis on tumorigenicity were explored *in vivo*.

**Results:**

Suppression of SNHG1 suppressed the viability, migration, and invasion but promoted apoptosis of FaDu cells *in vitro* (*P* < 0.01). PARP6 is a target of SNHG1, which was upregulated by SNHG1 knockdown in FaDu cells (*P* < 0.01). SNHG1 suppression and RARP6 overexpression inhibited FaDu cell proliferation, migration, and invasion (*P* < 0.05). SNHG1 suppression and RARP6 overexpression also inhibited tumorigenicity of HSCC *in vivo*. Furthermore, the protein expression of E-cadherin was significantly increased and that of N-cadherin, *β*-catenin, and XRCC6 was dramatically decreased in HSCC after SNHG1 suppression or/and RARP6 overexpression both *in vitro* and *in vivo* (*P* < 0.01).

**Conclusions:**

SNHG1 silencing inhibits HSCC malignant progression via upregulating PARP6. XRCC6/*β*-catenin/EMT axis may be a possible downstream mechanism of the SNHG1/PARP6 axis in HSCC. SNHG1/PARP6 can be used as a promising target for the treatment of HSCC.

## 1. Introduction

Head and neck squamous cell carcinoma (HNSCC) comprises a group of common solid tumors occurring in the squamous epithelium of the oral cavity, oropharynx, larynx, and hypopharynx [1]. Among HNSCC, hypopharyngeal squamous cell carcinoma (HSCC) is an aggressive cancer and has the worst prognosis [2]. Despite advances in surgical resection, neoadjuvant chemotherapy, and radiation therapy, the 5-year survival rate of patients with HSCC is only 25% to 40% [3]. Therefore, elucidation of key molecular mechanisms has great importance to improve the clinical outcomes of HSCC.

Long noncoding RNAs (lncRNAs) have been found to function as key regulators in cancers. lncRNAs are a group of RNAs with lengths of more than 200 nucleotides but lack protein-coding ability [4]. Increasing studies have revealed that lncRNAs exhibit diverse roles in many physiological and pathological processes [5–7]. For example, lncRNA urothelial carcinoma-associated 1 (UCA1) has an oncogenic role in HSCC, and high UCA1 expression is associated with worse prognosis [8]. Blocking lncRNA MALAT1 can restrain the development of laryngeal and hypopharyngeal carcinoma [9]. Identification of crucial lncRNAs can help elucidate the pathogenesis of HNSCC. lncRNA Small Nucleolar RNA Host Gene 1 (SNHG1), located at chromosome 11q12.3, reportedly plays an oncogenic role in diverse cancers, such as colorectal [10], breast [11], and cervical cancers [12]. SNHG1 also can promote memory formation while impeding effector CD8 in acute viral infections including COVID-19 [13]. In ovarian cancer, SNHG1 stimulates tumor progression by enhancing cancer cell epithelial-mesenchymal transition (EMT) and invasiveness [14]. SNHG1 silencing exerts the tumor-suppressive effect in breast cancer [15, 16]. Besides, SNHG1 knockdown prevents tumor growth and metastasis of hepatocellular carcinoma [17]. Particularly, SNHG1 is involved in the regulation of oral squamous cell carcinoma [18], laryngeal squamous cell carcinoma [19], and esophageal squamous cell cancer [20]. However, the role of SNHG1 in HSCC has not been reported.

lncRNAs also act as critical regulators of gene expression in a variety of human cancers [21, 22]. SNHG1 promotes the proliferation of gastric cancer cells via increasing DNMT1 expression [23]. SNHG1 actions as an oncogenic role in breast cancer through regulating LMO4 expression [24]. Poly (ADP-ribose) polymerase 6 (PARP6) belongs to the PARP family, which plays a crucial role in numerous cancers, such as gastric [25] and colorectal adenocarcinoma [26] and breast cancers [27]. However, the function of PARP6 in HSCC development is largely unknown. Whether SNHG1 contributes to HSCC via regulating PARP6 has not been reported.

In the present study, the effects and possible regulatory mechanisms of SNHG1 on the malignant phenotypes of HSCC cells were investigated *in vitro* and *in vivo*. These findings provide a new perspective for the development of therapeutic strategies for HSCC.

## 2. Materials and Methods

### 2.1. Cell Culture

A human HSCC cell line (FaDu) was obtained from American Type Culture Collection (Manassas, VA, USA). Cells were cultured in Dulbecco's modified Eagle medium (DMEM) containing 10% fetal bovine serum (FBS, Gibco, Sydney, Australia) and 1% penicillin-streptomycin in a 37°C incubator filled with 5% CO_2_ atmosphere.

### 2.2. Cell Transfection

Short hairpin RNAs targeting SNHG1 (sh1-SNHG1 and sh2-SNHG1) and shRNA negative control (sh-NC) were synthesized by Hanbio Co. Ltd. (Shanghai, China). FaDu cells (70%–80% confluence) were transfected with 30 nM sh-NC, sh1-SNHG1, or sh2-SNHG1 using Lipofectamine RNAiMax (Invitrogen, Carlsbad). In addition, to overexpress Poly (ADP-ribose) polymerases 6 (PARP6), FaDu cells were transfected with lentiviral constructs containing PARP6 (lenti-PARP6). Cells were harvested after 48 h posttransfection. Transfection was confirmed by measuring the mRNA expression of SNHG1 and PARP6 using the quantitative reverse-transcription PCR (qRT-PCR) assay.

### 2.3. qRT-PCR

The Trizol reagent (Invitrogen) was used for extracting total RNA from FaDu cells in different groups. cDNA synthesis was conducted by reverse-transcription reactions using the PrimeScriptTM RT Master Mix Kit (Takara, Japan). For detection of gene expression, qRT-PCR was then carried out using an SYBR Premix Ex Taq kit (TaKaRa, Japan) on the Rotor-Gene RG-3000A (Corbett Life Science, Sydney, Australia). Conditions for PCR were 95°C for 10 min, followed by 45 cycles of 95°C for 15 s and 60°C for 60 s. U6 and GAPDH were used as internal controls for miRNAs and RNAs, respectively. Relative expression of specific genes was then determined using the 2^−ΔΔCt^ method.

### 2.4. CCK-8 Assay

FaDu cells were collected, centrifuged, and resuspended with a fresh complete medium. FaDu cells were seeded into a 96-well plate (2 × 10^3^ cells/well) for 0, 24, 48, and 72 h. Then, 10 *μ*L CCK-8 solution (Beyotime, Jiangsu, China) was incubated with cells in each well for 2 h at 37°C with 5% CO_2_. The absorbance value (OD 450 nm) was detected using a microplate reader (Bio-Rad, Hercules, USA).

### 2.5. Transwell Assay

Cell migration and invasion were determined using Transwell assays. Different from the migration assay, the upper chamber of the Transwell insert (8 mm pore size; Millipore, Billerica, MA, USA) was precoated with Matrigel for invasion assay. In brief, FaDu cells (1 × 10^6^/mL) in different groups were resuspended with serum-free media, 200 *μ*L of which was added into the upper chamber containing serum-free medium. Meanwhile, 600 *μ*L of the complete medium with 20% FBS was added into the lower chamber. After incubating at 37°C for 24 h, cells on the lower membrane were fixed with formaldehyde for 30 min and stained with 0.1% crystal violet for 20 min. Cells in five randomly selected fields under a 400x magnification were observed under an IX71 inverted microscope (Olympus, Tokyo, Japan).

### 2.6. Flow Cytometry

FaDu cells (1 × 10^6^/mL) in different groups were digested with 0.25% trypsin and resuspended in a 300 *μ*L binding buffer. Following the manufacturer's protocol of the Annexin V-FITC Apoptosis Detection Kit (Beyotime), cells were double-stained with 5 *μ*L Annexin V-FITC for 15 min and then with 10 *μ*L propidium iodide (PI) for 10 min in the dark. Apoptotic cells were detected using a FACSCalibur flow cytometer (BD Biosciences, Mountain View, CA) with CELL Quest software (BD Biosciences).

### 2.7. Western Blot Assay

Total protein extraction from FaDu cells was performed by lysing with RIPA lysis buffer (Beyotime). After determining the protein concentrations using a BCA Protein Assay Kit (Thermo Scientific, Waltham, USA), protein extracts (50–100 *μ*g per lane) were separated on 12% SDS-polyacrylamide gels and transferred onto polyvinylidene fluoride (PVDF) membranes (Millipore, Billerica, MA, USA). Immunoblotting was then performed using the primary antibodies, including anti-PARP6 (1 : 1,000, ab79640), anti-XRCC6 (1 : 2,000, ab233237), anti-*β*-catenin (1 : 5,000, ab32572), anti-E-cadherin (1 : 10,000, ab40772), anti-N-cadherin (1 : 5,000, ab76011), and anti-GAPDH (1 : 1,000, ab8245) (Abcam, Cambridge, UK), overnight at 4°C. The secondary antibody was a horseradish peroxidase-conjugated antibody (1 : 2,000, sc-2357, Santa Cruz Biotechnology, CA, USA). GAPDH was used as the control. Protein blots were visualized using Enhanced Chemiluminescence (ECL) kit (Thermo Scientific) and analyzed using Image J software (National Institutes of Health, USA). The method for western blotting was referred to as the previously described [28].

### 2.8. RNA Pull-Down Assay

Pierce TM Pull-Down PolyHis Protein: a Protein Interaction Kit (Pierce, USA) was used for RNA pull-down assay following the protocol of the manufacturer. In brief, sequences of SNHG1 were subjected to PCR amplification, RNA extraction, reverse-transcription into cDNA, transcription *in vitro*, and RNA purification. Purified RNA transcripts were then labeled with Biotin. Then, 1 mg cell lysates were incubated with biotinylated transcripts at 4°C for 1 h with rotation. Afterward, cell protein lysate was added with pierce nucleic acid compatible streptavidin magnetic beads to sediment the RNA-protein complex. After washing the beads three times, proteins were retrieved by being boiled in 5× SDS-PAGE loading buffer and then subjected to western blot analysis.

### 2.9. RNA Immunoprecipitation (RIP)

The binding of SNHG1 and PARP6 was detected using RNA-Binding Protein Immunoprecipitation Kit (Millipore, Billerica, MA, USA). Followed by preparation of cell lysates, magnetic beads were conjugated with human anti-PARP6 (Millipore), which was used to enrich SNHG1 and PARP6. Normal Anti-IgG (Millipore) was utilized as a negative control. Immunoprecipitation and RNA purification were carried out for qRT-PCR analysis.

### 2.10. *In Vivo* Experiments

Animal experiments were approved by the Institutional Animal Care and Use Committee of The First Affiliated Hospital of Zhejiang Traditional Chinese Medical University. Four-week-old BALB/*c* mice (weighing 18–20 g, Shanghai Ling Chang Biological Technology Co., Ltd, Shanghai, China) were fed in sterilized cages (23 ± 1°C and 40–60% relative humidity under 12 h/12 h light/dark cycle) for 3 days with standard laboratory chow and adequate water. Animals were randomly divided into five groups, including model (control), lenti-NC, lenti-PARP6, sh-NC + lenti-PARP6, and sh-SNHG1 + lenti-PARP6 groups. For the observation of the tumourigenicity, 1 × 10^6^ FaDu cells transfected with sh-SNHG1, sh-NC, lenti-PARP6, and/or lenti-NC were injected subcutaneously into the right flank of nude mice. Animals in the model group were subcutaneously injected with the same volume of PBS. Tumor sizes of mice were measured every three days, followed by calculation of tumor volumes using the following formula: *V* (mm^3^) = (width^2^ × length) × 1/2. After 30 days, all mice were sacrificed by 70% CO_2_ asphyxiation followed by exsanguination. Tumor tissues in each group were weighed and frozen for subsequent experiments. All procedures were performed according to the protocols approved by the Institutional Animal Ethics Care and Use Committee.

### 2.11. TUNEL Assay

Tumors in different groups were cut into paraffin sections (4 *μ*m thick). Apoptosis in tumor samples was determined using the TUNEL assay (Beyotime). In brief, paraffin-embedded sections were subjected to deparaffining, hydration, and antigen retrieval. Afterward, the sections were covered with TUNEL detection solution, stained with streptavidin-HRP solution, and then visualized by incubation with diaminobenzidine (DAB). After redyeing with hematoxylin, sections were dehydrated, mounted, and observed under the microscope. The percentage of apoptosis was calculated as follows: apoptosis rate = (apoptotic cells/total cells) × 100%.

### 2.12. Statistical Analysis

All data are presented as the means ± standard deviation. The significant differences between groups were evaluated with one-way ANOVA. Further comparison between groups was performed by the post hoc Tukey test. Statistical analyses were conducted using the GraphPad Prism (version 7.0; GraphPad Software, La Jolla, CA, USA), and *P* < 0.05 indicated statistically significant.

## 3. Results

### 3.1. Suppression of SNHG1 Inhibited the Malignant Phenotypes of HSCC Cells

To explore the role of SNHG1 in HSCC cells, we knocked down the expression of SNHG1 in FaDu cells (a human HSCC cell line). As a result, SNHG1 expression was significantly (*P* < 0.01) decreased in both sh1-SNHG1 and sh2-SNHG1 groups compared to that in the sh-NC group, suggesting that SNHG1 expression was successfully suppressed in FaDu cells (Figure 1(a)). FaDu cell viability was significantly (*P* < 0.01) inhibited after suppression of SNHG1 (Figure 1(b)). Transwell assay revealed that suppression of SNHG1 resulted in dramatic decrease in the ratios of migrated and invaded FaDu cells, indicating that suppression of SNHG1 inhibited HSCC cell migration and invasion (*P* < 0.01, Figure 1(c)). The percentage of apoptotic cells in both the sh1-SNHG1 and sh2-SNHG1 groups was markedly increased compared to that in the sh-NC group (*P* < 0.01, Figure 1(d)), indicating that suppression of SNHG1 promoted HSCC cell apoptosis.

### 3.2. SNHG1 Directly Targeted PARP6 and Affected the Expression of XRCC6, *β*-Catenin, and EMT-Related Proteins

To investigate the relationship between SNHG1 and PARP6, RNA pull-down and RIP assays were conducted. Consistent results were obtained that SNHG1 could directly target PARP6 (Figures 2(a) and 2(b)). Moreover, western blotting confirmed that suppression of SNHG1 significantly (*P* < 0.01) promoted the protein expression of PARP6 (Figure 3). To further explore the possible downstream mechanism, the protein expression of XRCC6, *β*-catenin, and EMT-related proteins (E-cadherin and N-cadherin) was detected. The results showed that suppression of SNHG1 significantly (*P* < 0.01) promoted the E-cadherin level but inhibited the expression of N-cadherin, *β*-catenin, and XRCC6 (Figure 3).

### 3.3. Overexpression of PARP6 Enhanced the Inhibitory Effects of SNHG1 Suppression on HSCC Cells

To further confirm whether PARP6 was a target of SNHG1, PARP6 was overexpressed in FaDu cells by lentivirus infection. Results showed that expression of PARP6 was markedly increased after overexpression of PARP6, which was further elevated by sh-SNHG1 addition (*P* < 0.01, Figure 4(a)). Moreover, compared to the control group, overexpression of PARP6 significantly (*P* < 0.05) inhibited cell viability, migration, and invasion and facilitated cell apoptosis (Figures 4(b)–4(d)). Moreover, compared to the lenti-PARP6 group, overexpression of PARP6 and suppression of SNHG1 had synergistic effects in inhibiting the malignant phenotypes of HSCC cells (*P* < 0.05, Figures 4(b)–4(d)). These data confirmed that PARP6 was a functional target of SNHG1 to regulate the development of HSCC. Furthermore, we found that the protein expression of PARP6 and E-cadherin was remarkably increased, whereas that of N-cadherin, *β*-catenin, and XRCC6 was dramatically decreased after overexpression of PARP6, which were further decreased after sh-SNHG1 addition (*P* < 0.01, Figure 5).

### 3.4. SNHG1/PARP6 Axis Regulated Tumorigenicity of HSCC *In Vivo*

The effects of the SNHG1/PARP6 axis on tumorigenicity were further investigated *in vivo*. The results showed that the tumor size and volume were significantly (*P* < 0.01) decreased in lenti-PARP6 xenografts or sh-SNHG1 + lenti-PARP6 xenografts compared to those in the model (control) group (Figure 6(a)). TUNEL assay showed that tissue apoptosis was markedly promoted after overexpression of PARP6 alone or with suppression of SNHG1 (Figure 6(b)). Moreover, the protein expression of PARP6 and E-cadherin was significantly (*P* < 0.01) increased, whereas that of N-cadherin, *β*-catenin, and XRCC6 was dramatically decreased in mice of the lenti-PARP6 group and the expression changes of these proteins were more obvious in mice in sh-SNHG1 + lenti-PARP6 group (*P* < 0.05Figure 7). These data indicated the role and possible mechanism of the SNHG1/PARP6 axis in tumorigenicity *in vivo*.

## 4. Discussion

Extensive studies have been devoted to exploring the role of lncRNAs in disease development, but it still needs further exploration. SNHG1 is an oncogenic lncRNA controlling cancer progression, upregulation of which is closely associated with advanced tumor stage, tumor size, TNM stage, and decreased overall survival [29]. Knockdown of SNHG1 inhibited cell proliferation, migration, and invasion but promoted cell apoptosis in laryngeal squamous cell carcinoma [19]. Consistently, we found that suppression of SNHG1 inhibited these malignant phenotypes of HSCC cells *in vitro* and *in vivo*, confirming that SNHG1 may play an oncogenic role in HSCC. Moreover, suppression of SNHG1 could target and upregulate the expression of PARP6. SNHG1/PARP6 affected the expression of XRCC6, *β*-catenin, and EMT-related proteins, suggesting SNHG1 may contribute to HSCC via binding to PARP6. These data may provide a new insight into the development of targeted therapy for HSCC.

PARP family is a class of multifunctional nuclear proteases that regulates multiple molecular events, such as intracellular DNA repair, cell cycle progression, gene transcription, and cell death [30, 31]. Moreover, the PARP family is involved in the genesis and development of various diseases, including tumors [32, 33]. Inhibition of PARP affects the radiosensitization of human papillomavirus (HPV)/p16-positive HNSCC cell lines [34]. PARP6 is a member of the PARP family, which is a tumor suppressor in colorectal cancer [35, 36]. Tang et al. demonstrated that PARP6 inhibits the metastasis and proliferation of hepatocellular carcinoma [37]. A report on breast cancer indicated that PARP6 can directly target ADP-ribosylate Chk1, leading to the multipolar spindle formation and apoptosis induction [27]. RNA pull-down and RIP assays revealed that SNHG1 could directly target PARP6 in HSCC cells. Moreover, overexpression of PARP6 inhibited proliferation, migration, and invasion of FaDu cells but promoted cell apoptosis. Collectively, we speculated that PARP6 may act as a tumor suppressor in HSCC, which is a functional target of SNHG1.

In addition, PARP6 reportedly inhibits XRCC6 expression by inducing degradation and thus affects the Wnt/*β*-catenin signaling pathway, leading to the suppression of hepatocellular carcinoma [37]. XRCC6, a gene coding Ku70 protein, is involved in DNA recombination and repair [38]. Aberrant expression of XRCC6 is implicated in development of several types of tumors, such as osteosarcoma [39] and cancers of digestive system [40]. Overexpression of XRCC6 has been found in a large cohort of HNSCC patients [41] as well as HNSCC cell lines [42], suggesting the important role of XRCC6 in HNSCC. We found that the protein expression of XRCC6 was dramatically decreased in HSCC cells after suppression of SNHG1, which was further enhanced after overexpression of PARP6. Therefore, we speculated that the SNHG1/PARP6 axis may contribute to HSCC development via targeting XRCC6.

Furthermore, XRCC6 is a regulator of the *β*-catenin/Wnt signaling pathway [39]. A Wnt/*β*-catenin signaling pathway is a key downstream mediating the role of PCDH20 in HSCC [43]. Wnt/*β*-catenin signaling pathway has a profound role in EMT progression [44]. SRY-related high mobility group box 9 (SOX9) promotes EMT via activating the Wnt/*β*-catenin pathway, which is achieved by the nuclear translocation of *β*-catenin [45]. EMT, an early event of tumor metastasis, is characterized by the downregulation of E-cadherin (epithelial cell markers) and the upregulation of N-cadherin (mesenchymal cell markers) [46, 47]. EMT is implicated in the metastasis of HPV-negative pharyngeal squamous cell carcinoma [48]. In our *in vitro* and *in vivo* studies, the expression of E-cadherin was significantly increased and N-cadherin and *β*-catenin levels were dramatically decreased in HSCC cells after SNHG1 suppression or/and PARP6 overexpression. These data indicated that the *β*-catenin/EMT axis was a downstream mechanism of the SNHG1/PARP6 axis in HSCC.

## 5. Conclusion

Our findings reveal that SNHG1 is a key regulator in HSCC and may contribute to tumor development via targeting PARP6. XRCC6/*β*-catenin/EMT axis may be a possible downstream mechanism of the SNHG1/PARP6 axis in HSCC. SNHG1/PARP6 could be used as a promising biomarker or target for monitoring and treatment of HSCC.

## Figures and Tables

**Figure 1:** Suppression of SNHG1 inhibited the malignant phenotypes of hypopharyngeal squamous cell carcinoma (HSCC) cells. (a) qRT-PCR showed the SNHG1 expression in HSCC cell line (FaDu) by normalizing to GAPDH. (b) CCK-8 assay showed the FaDu cell viability. (c) Transwell assay revealed FaDu cell migration and invasion. (d) Flow cytometry showed FaDu cell apoptosis. FaDu cells were transfected with sh-NC, sh1-SNHG1, or sh2-SNHG1. Data are expressed as mean ± standard deviation (SD) (*n* = 3). ^*∗∗*^*P* < 0.01, compared with sh-NC.

**Figure 2:** The target relationship between SNHG1 and PARP6 in HSCC cells. (a) RNA pull-down and (b) RNA immunoprecipitation (RIP) assay to detect the binding of SNHG1 and PARP6 in FaDu cells. Data are expressed as mean ± SD (*n* = 3). ^*∗∗*^*P* < 0.01, compared with anti-IgG.

**Figure 3:** The expression of PARP6, XRCC6, *β*-catenin, and EMT-related proteins (E-cadherin and N-cadherin) in HSCC cells by western blot assay. FaDu cells were transfected with sh-NC, sh1-SNHG1, or sh2-SNHG1. Data are expressed as mean ± SD (*n* = 3). ^*∗∗*^*P* < 0.01, compared with sh-NC.

**Figure 4:** SNHG1/PARP6 axis inhibited the malignant phenotypes of HSCC cells. (a) qRT-PCR showed PARP6 expression in FaDu cells. (b) CCK-8 assay showed FaDu cell viability. (c) Transwell assay revealed FaDu cell migration and invasion. (d) Flow cytometry showed FaDu cell apoptosis. FaDu cells were transfected with lenti-NC, lenti-PARP6, sh-NC, or/and sh-SNHG1. Data are expressed as mean ± SD (*n* = 3). ^*∗∗*^*P* < 0.01, compared with lenti-NC. ^#^*P* < 0.05 and ^##^*P* < 0.01, compared with sh-NC + lenti-PARP6 group.

**Figure 5:** SNHG1/PARP6 axis affected the protein expression of XRCC6, *β*-catenin, and EMT-related proteins (E-cadherin and N-cadherin) in HSCC cells by western blot assay. FaDu cells were transfected with lenti-NC, lenti-PARP6, sh-NC, or/and sh-SNHG1. Data are expressed as mean ± SD (*n* = 3). ^*∗∗*^*P* < 0.01, compared with lenti-NC. ^##^*P* < 0.01, compared with sh-NC + lenti-PARP6 group.

**Figure 6:** SNHG1/PARP6 axis regulated tumorigenicity and tissue apoptosis of HSCC in vivo. (a) Tumor size and volume of differently treated mice (^*∗∗*^*P* < 0.01). (b) TUNEL showed tissue apoptosis of differently treated mice. BALB/*c* nude mice were subcutaneously injected with FaDu cells that were transfected with lenti-NC, lenti-PARP6, sh-NC, or/and sh-SNHG1. Data are expressed as mean ± SD (*n* = 5).

**Figure 7:** Effects of SNHG1/PARP6 axis in the expression of PARP6, XRCC6, *β*-catenin, and EMT-related proteins (E-cadherin and N-cadherin) in HSCC *in vivo*. Western blotting was used to detect the expression of PARP6, XRCC6, *β*-catenin, E-cadherin, and N-cadherin in tumor tissues of differently treated mice. BALB/*c* nude mice were subcutaneously injected with FaDu cells that were transfected with lenti-NC, lenti-PARP6, sh-NC, or/and sh-SNHG1. Data are expressed as mean ± SD (*n* = 5). ^*∗∗*^*P* < 0.01, compared with the lenti-NC group. ^#^*P* < 0.05 and ^##^*P* < 0.01, compared with the sh-NC + lenti-PARP6 group.

## Data Availability

The data used to support the findings of this study are available from the corresponding author upon request.
